The article "An Intelligent Animation Interaction Design Algorithm Based on Example and Parameterization" was retracted in 2023. Reasons: unreliable results or conclusions; concerns about the data; concerns about the peer review; concerns about the citations.

# An Intelligent Animation Interaction Design Algorithm Based on Example and Parameterization

**DOI:** 10.1155/2022/6017254

**Published:** 2022-07-21

**Authors:** Yingquan Wang, Peng Han, Bo Yang

**Affiliations:** ^1^School of Arts, Qingdao Huanghai University, Qingdao, Shandong 266427, China; ^2^Qingdao Huanghai University, Qingdao, Shandong 266427, China; ^3^Department of Secrecy Archive and Screen Culture, Logistics University of PAPF, Tianjin 300300, China

## Abstract

Intelligent design for the animation interaction is very challenging and needs to be resolved on priority basis. If this design is based on smart learning based mechanism, then it will be more appropriate and effective. Therefore, based on the idea of process modeling, the concrete method is based on example modeling and parameterization, and the VC programming environment is the tool. Animated interactions are not counted. The animation parameterization in the sample animation software and its attribute information are calculated, and the principle and realization process of the new animation interaction design are given, as well as the calculation method and steps of each area of animation elements. The same interaction design pattern can be filled in different areas by using parametric methods. In practice, we have increased the diversity of animation interaction design. The method proposed in this paper can quickly and automatically generate a virtual animation design network according to the user's design ideas and can be controlled by the user in real time interactively, providing a good interface and a new way for the user to design animation environment modeling.

## 1. Introduction

Initially, the current advancement in the technology has led to the development and realization of the different systems for different application domains. These systems must be smart enough to make timely decisions which are assumed to be accurate and precise. These decisions would be more accurate and precise if artificial intelligence or computational based techniques have been adopted in the developmental process of the modeling and simulation as well. Parametric animation modeling has been increasingly popular in numerous sectors, including video watching and game production, since the 21st century. The most essential thing to remember when modeling parametric animation is to model parametric animation [1], since the mode of parametric animation has an impact on the visual effect of the animation. Traditional modeling software for large-scale parametric animation modeling is time-consuming and takes a lot of personnel and material resources. The parametric animation process modeling approach is a viable option. The idea of process modeling can be well applied in research, education, and entertainment industries [2, 3]. The main purpose of this paper is to model the idea in terms of a similar process. Using sample-based modeling methods and parametric technology, a set of parametric animation interaction design systems are established, and large-scale parametric animation styles are generated in real time.

The article "An Intelligent Animation Interaction Design Algorithm Based on Example and Parameterization" was retracted in 2023. Reasons: unreliable results or conclusions; concerns about the data; concerns about the peer review; concerns about the citations.

This paper proposes an example-based animation interaction design algorithm. Through the extraction of animation interaction point attribute information [4, 5], the original animation style characteristics are maintained to a certain extent, and the average parameterization method is used to map the generated animation interaction to different animations in the area.

For animation interaction and animation modeling, the process modeling approach is employed. The L-system is used in the majority of existing approaches, and a fixed system is used to drive the model's progressive creation. It is frequently difficult to add new rules to manage the authenticity of the model due to the strictness and complexity of the rule system. The tensor field technique has recently been offered as a way to assist the design of animation interaction algorithms, although this method has flaws in algorithm transition. With the use of some existing data, example-based modeling technologies may swiftly develop more complicated models. Texture synthesis is where these approaches are most commonly applied, as evidenced by literature [6–8]. Reference [9] suggested a method for generating urban landscapes using sample GIS data, which obtained good results and realized regional transition and white natural connections.

The parametric method of mapping from one surface to another known area was first used for texture mapping. The parameterization process of this paper is based on the idea of the literature [10]. The coordinate mean method is used to express the coordinates of each two-dimensional point as a convex combination of its neighbor points, which is a method of harmonic mapping, which has both length and angle maintained to a certain extent [11, 12].

This article is dedicated to the development of an effective modeling technique or algorithm which is specifically designed for the interaction of the animations. This mechanism could be more impressive if artificial intelligence enabled designed and decision support systems have been developed. Actually, the proposed system is based on the example which is realized through the animation extraction of the point of interaction. Moreover, the proposed model or design has the built-in capacity to maintain various characteristics of the different styles.

The article "An Intelligent Animation Interaction Design Algorithm Based on Example and Parameterization" was retracted in 2023. Reasons: unreliable results or conclusions; concerns about the data; concerns about the peer review; concerns about the citations.

The remainder of the paper is organized as follows.

The rationale for parameterized implementation with examples is reported in the second section of the paper along with various parameters which are described in the paper. Parametric animation interaction design algorithm and its various steps along with detailed discussion are presented in the third section of the paper. Parametric animation interaction design isdiscussed in detail in the fourth section of the paper which is followed by the conclusion section.

## 2. Rationale for Parameterized Implementation with Examples

A typical structure-hinge four-bar mechanism is taken as an example to illustrate the design method of parametric animation.

(1) Determining the parameters that need to be changed: As shown in Figure 1, showing the four-bar mechanism ABCD, the parameters that need to be changed are the length L of the rod AB, the length L2 of the BC, the length L3 of the CD, and the length L4 of the AD [13]. At the same time, from the perspective of control, the speed of animation playback is also an adjustable parameter, and its factor is set to L7.
(2) Determining the overall framework: control of four variable parameters and data display, animation playback, playback control and speed control, the conversion relationship between the size of the animation area and the length of the four rods, and so forth [14]. The overall frame of the four-bar mechanism is shown in Figure 2. The conversion relationship between the size of the animation area and the length of the four rods can be based on the screen resolution.
(3) Programming, including the following:
  1. The dynamic generation of the mechanism;
  2. The control of parameter dragging;
  3. Other judgment knowledge related to the mechanism (whether it is composed of a mechanism, the basic type of the mechanism) and so on. The basic method is to find the coordinates of the four points *A*, *B*, *C*, and *D* and then connect the four points with a line.
(4) As shown in Figure 1, the four points *A*, *B*, *C*, *D* are put as symbols into the scene as Move-Clip, named AA, BB, CC, and DD, respectively. Among them, AA is fixed and used as the positioning reference, and the corresponding layer is established for easy control. The key lies in the action layer, as shown in Figure 3.
(5) Initialization preparation and related knowledge preparation. For the four-bar structure, the key lies in whether the four-bar structure is formed at any length and the basic type of the four-bar structure. Frame 1 of the action layer mainly does this work.

The main code on frame 1 of the action layer is as follows:

- Initial data preparation:
- Define variables: initial length of four rods _ global.11 = 50; _ global.12 = 90; _ global. 13 = 180; _ global. 14 = 180;
- animation initial speed variable_ global.17 = 1;
- Four-bar length dynamic display variable 111 = _ global. 11; 112 = global. 12; 113 = global. 13; 114 = _ global. 14, the four values are realized with dynamic text boxes combined with variables.
- The initial position of the graphic base reference point position: root.AA._ *x* = 200;
- root.AA..*y* = 250;
- scrollbar initial position_ giobal. Bar_ *x* = 538;
- //Adjust the basic reference point *X* position of the data drag slider;
- root.
- bar._*X* = _ global.bar._*x* + int((_ global.11–40
- 18)/1.4);
- *i* is the angle between AB and CD; *j* is the angle between CD and AD_ global.*i* = 
- 30; as shown in Figure 1.

The article "An Intelligent Animation Interaction Design Algorithm Based on Example and Parameterization" was retracted in 2023. Reasons: unreliable results or conclusions; concerns about the data; concerns about the peer review; concerns about the citations.

Function preparation:

global. Anguec can find the angle of *j* according to the angle of *i*, _global. Arguec = function(*q*) {.....
global arguei The angle of *i* can be found according to the angle of *j*, _global. Arguei = function(*q*) ......
global. Okj = function() ...... } judgment
global.arbitate = function(a, *b*, *c*, d) {//This function judges the length of the four-bar and returns the corresponding value
gmin = Math.min (Math.min(*a*, *b*), Math.min(*c*,*d*)); //Find the minimum of the four values
gmax = Math.max (Math.max(*a*, *b*), Math.max(*c*, *d*)); //Find the maximum of the four values
if(gmin + gmax< =*a*+*b* + *c* + d- (gmin + gmax)){//The sum of the minimum rod and the maximum rod is less than or equal to the sum of the other two rods;
if((*a* = = *c*)&&(*b* = = *d*)) { return 4; //If *a* = *c* and
*b* = *d*, must be “parallel double crank mechanism”}
if(*d* = gmin) {return2; //When the shortest rod is used as the frame, it must be a “double crank mechanism”}
f(*a* = = gmin |I *c* = = gmin) {return 1; //Take the adjacent rod of the shortest rod as the frame, which must be “crank rocker mechanism”}
if(*b* = = gnin) {return 3; //When the opposite pole of the shortest pole is used as the rack, it must be a “double rocker mechanism”}}
else//When the Grashof discriminant is not satisfied, it must be a “double rocker mechanism” or a group not, a four-bar mechanism
{f((_ global.11 +_ global.12+ - global.13 > _ global.
14)&&(_ global.11 + - global. 12+- global. 14>_ global. 13)&(_ global. 11 +_ global. 14+_ global. 13 > _ global. 12) &&(_ global .14+_global.12+- global.13>- gobal.11))
{return 3; }
else return 5; }}

Calculate the coordinates of each point and use the line drawing function to draw the mechanism. Frame 2 of the action layer mainly does this work.

- root.createEmptyMovieClip(“me”, 1); //Dynamic creation
- MovieCip, so that the drawing function can be used.
- result = _ global. Arbitrate(_ global. 11, _ global. 12, _ glob-
- al. 13,_ global. 14); //This function returns the result according to the length of the four bars.
- if(result: = 1){
- type = “crank-rocker mechanism”;
- A global.*j* = - global. Arguecl(_. Global. *i*); //The following calculation B,
- The coordinates of points C and *D*;
- _root.BB._*x* = Math.cos(Math.PI/180*∗*._global.i) *∗*_
- global.11+ - root.AA._x;
- _root., BB._ *y* = _ root.AA._ y− Math. Sin(Math. P/180*∗*
- a global.i) *∗* - global.11;
- _root.DD._*x* = _root.AA._*x* + ._global.14;
- _ root.DD._ *y* = - root.AA. a *y*;
- _root.CC._*x* = _root.DD._*x* + Math.co8(Math.PI/180*∗*
- global.j)*∗*_ global.13; _ root.CC._ *y* = _ root.DD._ y- Math. sin(Math. PI/180
- a global.j) *∗*_ global.13;
- //below is the line drawing
- root.me.clear();
- with (_ root. me) {
- lineSty]e(4,0 × 330099, 100);
- moveTo(_ root. DD. _ *x*,_ root. DD. _ *y*); lineTo(_ root. CC._ *x*,_ root. CC._ *y*);
- lineStyle(2,0 × 339900, 100);
- moveTo(_ root.AA._ *x*,_ root.AA._ *y*);.
- lineTo(_ root.BB._ *x*,_ root.BB._ *y*);
- lineSyle(2,xefOf, 100);
- (xi) lineTo(_ root.CC._ *x*,_ root.CC._ *y*);
- (xii) }}
- (xiii) } This draws the four-bar mechanism.

The article "An Intelligent Animation Interaction Design Algorithm Based on Example and Parameterization" was retracted in 2023. Reasons: unreliable results or conclusions; concerns about the data; concerns about the peer review; concerns about the citations.

Dynamically change the lengths of the four rods, and display them, borrow the work of the second frame, and draw the mechanism. The third frame of the action layer mainly completes this work.

- //The following code refreshes the parameter value
- if(_ global. change = true) {
- 111 = _g]obal.11;
- 112 = ._g]obal.12;
- 113 = ._g]obal.13;
- 114 = _- global. 14;
- global.change = false;
- //Recalculate the position of each point ......
- if(_ global.*i*≥360) {_ global.*i* = 0; } if rod AB turns - a
- week, keep turning.
- _global.*i*+ = _global.17; //The angle rotated by the rod AB each cycle,
- Namely speed control, 17 is the change factor.
- } Drag the slider to change the action of the parameter. As shown in Figure 3, with the length of AB
- Take degree L1 as an example. Add the following code to the slider:
- onClipEvent(load) {
- top = this._*y*;
- left = ._global.LEFT;
- night = _ g]obal. RICHT:
- bottom = this._*y*;
- onClipEvent(enterFrame) {
- if(dragging = = true) {
- *r* = this._X - left;
- }}
- Double-click the slider to enter the button-level editing. As shown in Figure 2, add the following code:
- on(res){
- dragging = true;
- startDrag(““, false, left, top, right, bottom);
- root.stop();
- barx = _root.bar._x;
- on (release, releaseOutside){
- stopDrag();
- dragging = false;
- startDrag(“/cursor”, tue);
- global.11 = int((_ root. Bar1._ *x*-_ global. Bar_ *x* + 
- 18)*∗*1.4)  +  40;
- global.change = tue; }
- }
- }

Let the sample and parameterized animation move, and make speed control. Frame 4 of the action layer mainly does this work. In fact, the program is between 3 and 4 frames. Repeatedly loop. Action code is gotoAndPlay(3). At this point, the program design is completed. In order to ensure the continuous and smooth animation, the default 12 fps (12 frames per second) can be changed to 30∼50 fps during development [15]. The animation interaction design algorithm has passed the debugging of the above program, and the program is very suitable for online communication. If the animation is designed with frame animation, the parameters are fixed and cannot be changed.

The article "An Intelligent Animation Interaction Design Algorithm Based on Example and Parameterization" was retracted in 2023. Reasons: unreliable results or conclusions; concerns about the data; concerns about the peer review; concerns about the citations.

## 3. Parametric Animation Interaction Design Algorithm

In actuality, the majority of animation interactions are not linear. The sample model generated by the mouse is supplied as a straight-line segment for the designer's convenience, and then the system “curves” it, that is, replaces it with a continuous polyline segment [16, 17]. The steps are as follows (Algorithm 1). The starting point and end point of the input straight-line segment are src and dst, respectively, the length of the polyline segment is *d*_*SAMPLE*_, and the sampling angle range is *θ*_DEV_. These parameters can be set by the user. See the algorithm for the main steps.

The first-level area division is to find the closed part formed between animation interaction and boundary and between sample and boundary. Algorithms for computing interactions in graph theory are employed.

### 3.1. Secondary Animation Interaction Design Growth Algorithm

The user decides the mode of each animation interaction design area in the first-level animation interaction design area, and the system generates the second-level animation interaction design using different animation interaction design generation algorithms. Create an animation interaction design connection strategy and parameterization approach between distinct sections so that the secondary animation interaction design is both aesthetically beautiful and dynamic [18].

For each animation interaction design intersection v_*i*_, the attribute information we need to obtain or calculate includes two-dimensional coordinate information (*a*, *b*, *c*, *d*) in the image.

Levels *h*_*a*_ and *h*_*b*_ of the two streets pass through *v*_*i*_ (assuming at most two streets pass through each intersection, and each street is represented by a continuous polyline segment).

On each street passing through *v*_*i*_, the lengths of adjacent road segments have a mean of *μ*_*d*_ and a variance of *σ*_*d*_^2^.

On each street passing through *v*_*i*_, the mean *μ*_*a*_ and variance *σ*_*a*_^2^ of the angle are formed by adjacent road segments.

The article "An Intelligent Animation Interaction Design Algorithm Based on Example and Parameterization" was retracted in 2023. Reasons: unreliable results or conclusions; concerns about the data; concerns about the peer review; concerns about the citations.

### 3.2. Connection of Animation Interaction Design Area

Since the secondary animation interaction design is generated separately in each area, there may be inconsistencies at the boundary of adjacent areas [19]. For this reason, all animation interaction design algorithms in our adjacent areas that intersect the same area boundary are carried out. For judgment, merge the intersections that are too close, so that the animation interaction design between regions can be naturally connected.

The schematic diagram of the traversal algorithm is given, in which probability *p* is a binary Gaussian distribution function, and the specific form is given by formula (1), where *μ*=(*μ*_*a*_, *μ*_*d*_)^*T*^ is the mean and ∑ is the covariance matrix.

(1) $$\begin{array}{c} p\left(x\right)=\frac{1}{{\left(2\pi \right)}^{\text{d}ο}{\left|\sum \right|}^{1.2}}\exp\left[-\frac{1}{2}{\left(x-\mu \right)}^{1}\sum^{-1}\left(x-\mu \right)\right]. \end{array}$$

It can be seen intuitively from formula (1) that the target node *v*_*j*_ with the highest probability found in each single-step traversal process has such properties; the design value between *v*_*i*_ and *v*_*j*_ is the attribute information *μa*^0^ closest to *v*_*i*_. The angle is formed by the animation interaction design segment to *v*_*j*_ and the previous segment. The attribute information *μd*^1^ closest to *v*_*i*_ is an application example of the traversal algorithm. Among them, the input animation sample is a new animation interaction design generated, and the modeling result maintains the style of the original road to a certain extent.

## 4. Animated Interaction Design Parametric

The parameterization method used in this article refers to the idea of mean parameterization proposed in the literature. First, all the animation interaction design intersection points in the sample are triangulated, and then each vertex is represented as a convex combination of its neighbour nodes, as in formula (2), where the weight coefficient is calculated according to (4) and (5), and formula (2) satisfies the identity relationship of formulas (2) and (3). The mapping topology in the new animation interaction design technique is created using the matrix calculation method after listing the relational equations between the intersection locations, and the parameterized result is presented.

(2) $$\begin{array}{c} \sum_{i=1}^{k}\lambda_{i}v_{i}=v_{0}, \end{array}$$

(3) $$\begin{array}{c} \sum_{i=1}^{k}\lambda_{i}=1, \end{array}$$

(4) $$\begin{array}{c} \lambda_{i}=\frac{\omega_{i}}{\sum_{\int =1}^{k}\omega_{j}}, \end{array}$$

(5) $$\begin{array}{c} \omega_{i}=\frac{\tan\left(\alpha_{i-1}/2\right)+\tan\left(\alpha_{i}/2\right)}{\left\|v_{i}-v_{o}\right\|}. \end{array}$$

The article "An Intelligent Animation Interaction Design Algorithm Based on Example and Parameterization" was retracted in 2023. Reasons: unreliable results or conclusions; concerns about the data; concerns about the peer review; concerns about the citations.

### 4.1. Calculation of Animation Interaction Design Area

The calculation process of the second-level animation interaction design area is basically similar to the first-level animation interaction design area. These animation interaction designs are further subdivided to obtain the third-level animation interaction design and sample data. When subdividing, we consider the two following practical situations. All animation interaction designs have at least multi-instance support and parametric scale. Animation interaction design traces are mostly represented by polygons, and most of them are quadrilaterals.

The main steps of the subdivision process are as follows: firstl is finding the most common probability data of the sample and parameterization and calculating the longer central axis; second is sample on the central axis and the two long sides of the bounding box, respectively, and the average sampling distance Pre-set, allowing the distance between the actual sampling points to float slightly on the basis of the average value; third is connecting the corresponding sampling points to form a three-level animation interaction design [20, 21]. Calculate the closed area to obtain each building footprint, and analyze the results of each algorithm data sample to obtain the corresponding animation interaction design.

In order to improve the controllability of the modeling process and make the modeling effect more realistic, the system has designed an interactive interface, and the designer can modify and adjust a series of parameters. Global parameters and operations include the density of animation interaction design and animation interaction design style or animation interaction design image. Local parameter operations include animation interaction design and algorithm adjustment at all levels, as well as the position movement of animation nodes, deletion, addition of new parameters, etc., and all editing operations can be performed in real time.

## 5. Conclusion

This work offers an animation interaction design algorithm based on example and parameterization, develops various design techniques for various animation interaction designs, and provides a legality diagnosis strategy as well as an animation division and calculation method for animation interaction. Modeling builds the groundwork and gives a solid user interface while also introducing a new concept in animation interaction design modeling. The following are typical design phases for parametric animation: Determine which parameters should be altered. Establish a conceptual structure, investigate parameter relationships, and then develop code. We have designed parametric animation according to this method in the sample and parametric animation interaction design algorithm and have received good results. Parametric animation is a very good method for learners to conduct self-inquiry learning, because there can be countless changes of this type, and each learner may see different things. From the perspective of actual teaching, it greatly improves learning. At the same time, with a little modification, it can be transformed into a parameter input-type interactive animation, which can turn the learner's thoughts into reality and achieve better learning and teaching effects.

The article "An Intelligent Animation Interaction Design Algorithm Based on Example and Parameterization" was retracted in 2023. Reasons: unreliable results or conclusions; concerns about the data; concerns about the peer review; concerns about the citations.

## Figures and Tables

**Figure 1:** A typical structure of animation interaction design method.

**Figure 2:** The overall framework of animation interaction design four-bar mechanism.

**Figure 3:** The basic type of action layer four-bar structure.

**Algorithm 1:** Parametric animation interaction design algorithm flow.

## Data Availability

The datasets used and analyzed during this study are available from the corresponding author upon reasonable request.
